# Feedback Delay of Sports Intelligent Learning System Based on Model Predictive Control

**DOI:** 10.1155/2022/5939421

**Published:** 2022-05-31

**Authors:** Haidong Lv

**Affiliations:** Physical Education Departmentof Shandong University (Weihai), Shandong, Weihai 264209, China

## Abstract

In this paper, a trajectory tracking controller based on linear time-varying model prediction is developed, and the model predictive control theory based on the six degrees of freedom dynamic model and tire model is applied. Combined with the soft constraint of turning angle and the control algorithm to ensure the stability, the trajectory tracking is realized. The terminal node is a wearable device. The terminal node is equipped with a pressure sensor and attitude sensor network to collect human data, and then the terminal node sends the data to the ZigBee network. The data in the sensor network will be received by the gateway, and the data will be processed and displayed on the PC software after being received by the gateway. Finally, the data is saved to the remote server for archiving. The application of intelligent learning systems in sports makes up for many shortcomings of traditional sports. The teaching of the course consists of seven types of intelligent courses, which not only conform to the spirit of high-quality education but also combine the shortcomings of traditional physical education learning and combines several intelligent theories and the need for time development. The purpose is to develop a new sports model suitable for students' all-round development. Under the guidance of the theory of intelligent learning system, this paper establishes a new and diverse movement model, including various educational models, educational contents, educational methods, student-based learning model, and multidimensional evaluation. By comparing and analyzing the results of the two groups, the multiple intelligences physical education is more suitable for the development of modern students' various intelligences. According to the physical education learning questionnaire, students also learn more methods and contents and accept diversified teaching evaluation, which expands the development direction of students.

## 1. Introduction

The model predictive control has a feedforward feedback structure, which makes it possible to process high-dimensional systems with multiple variables, multiple inputs, and multiple outputs, and can explicitly and actively deal with the hard constraints in the time domain for the purpose of optimization. Therefore, we have gained a lot of professional knowledge, and applications are gradually expanding beyond the field of industrial process control, including new applications such as high-speed dynamic systems and embedded systems. The solution of model predictive control is completed by repeating online calculation in a limited sampling time interval, not just an offline calculation. The new application field also has a higher demand for model predictive control. The demand is analyzed and an intelligent learning system is designed [1]. The terminal node equipment including wearable pressure measurement and joint activity measurement is developed. The wearable node has low power consumption and convenient data storage. Because the flash inside the wearable device is used to store data, there is no need to worry about data loss. At the same time, the corresponding upper computer is developed [2]. The PC can display the human data in real time through the sensor network and can also manage and set the wearable terminal node through the upper computer. Finally, the data is uploaded to the remote server in the sensor network to save the data, which is convenient for tracking and recording the data of the patient. At the same time, the system has the function of alarm and prompt. When the patient does not use the wearable device, the system will inform the patient [3]. The theory of intelligent learning system shows that each learning system has eight relatively independent intelligence, which are not isolated for our practice, study, and life. Especially in the physical education learning activities, only when the various intelligent learning systems are used in a complete, reasonable, close, and coordinated way, can we make more effective use of personal skills [4]. The basic course of school education is the physical education course, which is also the key point of school education. It plays an important role in training new and universal students and talents needed in modern society. At present, the education department in China is still in the stage of research and gradual improvement. In many places, educators need to find out problems, improve their education, and carry out comprehensive and thorough reform and construction of physical education [5]. The paper builds a new model of physical education based on the theory of multiple intelligence, which can further promote the development and progress of school physical education and the existing school physical education in China, and lay a foundation for reviewing learning objectives and educational achievements.

## 2. Related Works

This paper [6] introduces the delay feedback buck digital control converter. Based on the study of the control method and the principle of parameter adjustment, it not only verifies the software simulation but also verifies the effect of the control parameter value in the real object. It is different from the previous power circuit with the addition of op amp, voltage comparator, signal generator, and other analog circuits. To concentrate all the control parts on the digital controller, one is to solve the problem that analog circuit devices are difficult to change and adjust in real time, and the other is to provide a new idea and direction for the development of control. In the future, the control part will rely more on intelligent chip processing [7]. The development of chaos is introduced in the literature. From the emergence of chaos in various disciplines to the infiltration of chaos into nonlinear circuits, the previous research results and control methods in nonlinear circuits are briefly described. In this paper, the characteristics, analysis methods, and theoretical basis of chaos are introduced [8]. The stability of the buck converter at a fixed point is analyzed by discrete iteration. On this basis, the simulation circuit is built to study the chaos caused by the change of parameters. This paper focuses on the study of chaos control methods, analyzes and compares the advantages and disadvantages of different methods, deeply explores the mechanism of the delay feedback method, and adjusts the PID parameters when adding time delay, introduces the inverse Nyquist curve, and determines the proportional gain range, which is verified by simulation. In this paper, particle swarm optimization (PSO) is introduced to solve the optimization problem of finite model predictive control [9]. At the same time, through the study of the parallel computing structure of particle swarm optimization algorithm, the foundation of the parallel acceleration algorithm of FPGA hardware of the controller is established. With regard to the implementation of FPGA hardware, the hardware circuit is designed according to the parallel structure of the algorithm, which greatly improves the online computing ability of the controller so that the parallel computing structure of the hardware can be effectively used [10]. In this paper, the application of particle swarm optimization (PSO) to model predictive control (MPC) optimization is introduced, and the constrained PSO algorithm is proposed. We first show the principle and formula of the algorithm and then use the penalty function method to deal with the constraints [11]. Compared with the basic particle swarm optimization method, this algorithm can effectively deal with the constrained problem. Finally, we use linear and nonlinear algorithm examples to test the effectiveness of the constraint group method of model predictive control and compare and analyze the constraint group method with the general method to determine the computational power of the planning method [12]. According to the algorithm itself and the example algorithm, the selection principle of each optimization algorithm is summarized, which lays the foundation for the hardware implementation algorithm of model predictive control. This paper introduces two FPGA hardware methods to implement the model predictor. First of all, we propose how to implement SOPC embedded system based on FPGA. Nios II processor is built into an FPGA chip, and standard components are added to improve the hardware and software architecture of the SOPC system [13]. In order to make full use of the parallel computing function of FPGA, we develop a method to realize the complete hardware of FPGA and use the semiautomatic modular FPGA design method to design the controller. Through the combination of FPGA parallel computing and pipeline structure, the computing power of the MPC controller is enhanced. This method can improve computing performance, but it will consume more hardware resources.

## 3. Model Predictive Control and Sensor Network Model Design

### 3.1. Model Predictive Control

This chapter introduces the process of deriving the algorithm expression of linear time-varying model predictive control (ltv-mpc) and transforming the ltv-mpc optimization problem into a standard square programming (QP) problem which is easy to be solved by computer.

Consider the following discrete nonlinear systems:

(1) $$\begin{array}{c} \xi \left(t+1\right)=f\left(\xi \left(t\right),\mu \left(t\right)\right),\\ \xi \left(t\right)\in \chi ,\\ \mu \left(t\right)\in \Omega . \end{array}$$

Assuming that the origin of the system is *f*(0, 0) = 0, take this point as the control target of the system. For any *N* ∈ *Z*+, consider the following cost function:

(2) $$\begin{array}{c} J_{N}\left(\xi \left(t\right),U\left(t\right)\right)=\sum_{k=t}^{t+N-1}l\left(\xi \left(t\right),\mu \left(t\right)\right)+P\left(\xi \left(t+N\right)\right), \end{array}$$

The finite time domain optimization problem solved in each step is as follows:

(3) $$\begin{array}{c} \underset{U_{t},\xi_{t+1,t,\cdots \xi t+N\neq }}{\min}J_{N}\left(\xi \left(t\right),U\left(t\right)\right)=\sum_{k=t}^{t+N-1}l\left(\xi \left(t\right),\mu \left(t\right)\right)+P\left(\xi \left(t+N\right)\right),\\ \text{subj.to }\xi_{k+1,t}=f\left(\xi_{k,t},\mu_{k,t}\right)k=t,\ldots ,t+N-1,\\ \xi_{k,t}\in \chi k=t,\ldots ,t+N-1,\\ \mu_{k,t}\in \Omega k=t,\ldots ,t+N-1,\\ \xi_{t,t}=\xi \left(t\right),\\ \xi_{N,t}\in \chi_{f}. \end{array}$$

The difficulty of nonlinear model predictive control depends on the order of the state equation of the system. The greater the order of the system, the greater the difficulty. If the nonlinear system is linearized and the linear model predictive control algorithm is used to solve the problem, the calculation amount can be reduced and the calculation performance can be improved. The linearized system is determined by the time change and can be divided into two systems (linear time-invariant system and linear time-varying system) [14]. Linear time the invariant system has large control error and can not get enough track tracking control effect. Compared with solving nonlinear problems directly, the complexity of the calculation is significantly reduced, and the control accuracy is improved effectively compared with the linear time-invariant system.

### 3.2. Linear Time-Varying Model Predictive Control

Compared with nonlinear model predictive control, linear time-varying model predictive control has less computation and simpler resolution. This section will show how to convert a nonlinear system into a linear time-varying system.

(4) $$\begin{array}{c} {\hat{\xi }}_{0}\left(k+1\right)=f\left({\hat{\xi }}_{0}\left(k\right),{\hat{\mu }}_{0}\left(k\right)\right),\\ {\hat{\xi }}_{0}\left(0\right)\in \xi_{0},\\ {\hat{\mu }}_{0}\left(k\right)\in \mu_{0}. \end{array}$$

Carrying out the first-order approximate Taylor expansion, we get the following:

(5) $$\begin{array}{c} \xi \left(k+1\right)=f\left({\hat{\xi }}_{0}\left(k\right),{\hat{\mu }}_{0}\left(k\right)\right)+{\frac{\partial f}{\partial \xi }|}_{{\hat{\xi }}_{0}\left(k\right),{\hat{\mu }}_{0}\left(k\right)}\left(\xi \left(k\right)-{\hat{\xi }}_{0}\left(k\right)\right)+{\frac{\partial f}{\partial \mu }|}_{{\hat{\xi }}_{0}\left(k\right),{\hat{\mu }}_{0}\left(k\right)}\left(\mu \left(k\right)-{\hat{\mu }}_{0}\left(k\right)\right). \end{array}$$

Substituting it into the formula:

(6) $$\begin{array}{c} \xi \left(k+1\right)={\hat{\xi }}_{0}\left(k+1\right)+{\frac{\partial f}{\partial \xi }|}_{{\hat{\xi }}_{0}\left(k\right),{\hat{\mu }}_{0}\left(k\right)}\left(\xi \left(k\right)-{\hat{\xi }}_{0}\left(k\right)\right)+{\frac{\partial f}{\partial \mu }|}_{{\hat{\xi }}_{0}\left(k\right),{\hat{\mu }}_{0}\left(k\right)}\left(\mu \left(k\right)-{\hat{\mu }}_{0}\left(k\right)\right). \end{array}$$

Make the following settings:

(7) $$\begin{array}{c} A_{k,0}={\frac{\partial f}{\partial \xi }|}_{{\hat{\xi }}_{0}\left(k\right),{\hat{\mu }}_{0}\left(k\right)},\\ B_{k,0}={\frac{\partial f}{\partial \mu }|}_{{\hat{\xi }}_{0}\left(k\right),{\hat{\mu }}_{0}\left(k\right)},\\ \delta \xi \left(k+1\right)=\xi \left(k+1\right)-{\hat{\xi }}_{0}\left(k+1\right),\\ \delta \xi \left(k\right)=\xi \left(k\right)-{\hat{\xi }}_{0}\left(k\right),\\ \delta \mu \left(k\right)=\mu \left(k\right)-{\hat{\mu }}_{0}\left(k\right). \end{array}$$

(7) can be written as follows:

(8) $$\begin{array}{c} \delta \xi \left(k+1\right)=A_{k,0}\delta \xi \left(k\right)+B_{k,0}\delta \mu \left(k\right). \end{array}$$

(8) can be written as follows:

(9) $$\begin{array}{c} \xi \left(k+1\right)=A_{k,0}\xi \left(k\right)+B_{k,0}\mu \left(k\right)+d_{k,0}\left(k\right). \end{array}$$

### 3.3. Predictive Model Design

First consider the following nonlinear dynamic system:

(10) $$\begin{array}{c} \dot{\xi }\left(t\right)=f\left(\xi \left(t\right),\mu \left(t\right)\right),\\ \eta \left(t\right)=h\left(\xi \left(t\right),\mu \left(t\right)\right). \end{array}$$

Convert the nonlinear system into a linear time-varying system:

(11) $$\begin{array}{c} \xi \left(k+1\right)=A_{k,t}\xi \left(k\right)+B_{k,t}\mu \left(t\right)+d_{k,t},\\ \eta \left(t\right)=C_{k,t}\xi \left(k\right)+D_{k,t}\mu \left(t\right)+e_{k,t}, \end{array}$$

Correspondingly transform the data of the system state equation to obtain a new state space equation.

(12) $$\begin{array}{c} {\tilde{A}}_{k,t}=\left(\begin{array}{cc} A_{k,t} & B_{k,t}\\ 0_{m\times n} & I_{m} \end{array}\right),\\ {\tilde{B}}_{k,t}=\left(\begin{array}{c} B_{k,t}\\ I_{m} \end{array}\right),\\ {\tilde{C}}_{k,t}=\left(\begin{array}{cc} C_{k,t} & D_{k,t} \end{array}\right),\\ {\tilde{D}}_{k,t}=D_{k,t},\\ \tilde{\xi }\left(k|t\right)=\left(\begin{array}{c} \xi \left(k|t\right)\\ \mu \left(k-1|t\right) \end{array}\right),\\ \tilde{d}\left(k|t\right)=\left(\begin{array}{c} d\left(k|t\right)\\ 0_{m} \end{array}\right). \end{array}$$

A new state space expression can be obtained:

(13) $$\begin{array}{c} \tilde{\xi }\left(k+1|t\right)={\tilde{A}}_{k,t}\tilde{\xi }\left(k|t\right)+{\tilde{B}}_{k,t}\Delta \mu \left(k|t\right)+{\tilde{d}}_{k,t},\\ \eta \left(k|t\right)={\tilde{C}}_{k,t}\tilde{\xi }\left(k|t\right)+{\tilde{D}}_{k,t}\Delta \mu \left(k|t\right)+e_{k,t}. \end{array}$$

Among them,

(14) $$\begin{array}{c} \Delta \mu \left(k|t\right)=\mu \left(k|t\right)-\mu \left(k-1|t\right),\\ \xi \left(t|t\right)=\xi \left(t\right),\\ \mu \left(t-1|t\right)=\mu \left(k-1\right). \end{array}$$

The system output of the new state space equation can be calculated as follows:

(15) $$\begin{array}{c} \eta \left(k|t\right)={\tilde{C}}_{k,t}\overset{k-1}{\prod }{\tilde{A}}_{i,t}\tilde{\xi }\left(t|t\right)+\prod_{i=t}^{k-1}{\tilde{C}}_{k,t}\prod_{j=i+t}^{k-1}{\tilde{A}}_{j,t}\left[{\tilde{B}}_{i,t}\Delta \mu \left(i|t\right)+\tilde{d}\left(i|t\right)\right]+{\tilde{D}}_{k,t}\Delta \mu \left(k|t\right)+e\left(k|t\right). \end{array}$$

If the prediction time domain of the system is Hp and the control time domain is Hc, the following assumptions are made:

(16) $$\begin{array}{c} \Delta \mu \left(t+H_{c}|t\right)=\Delta \mu \left(t+H_{c}+1|t\right)=\ldots =\Delta \mu \left(t+H_{p}-1|t\right)=0. \end{array}$$

Among them,

(17) Yt=ηt+1tηt+2t⋮ηt+Hpt,Ψt=C˜t+1,tA˜t,tC˜t+2,tA˜t+1,tA˜t,t⋮C˜t+Hp,t∏ t+HP−1i=t−˜A˜i,t,Θt=C˜t+1,tB˜t,tD˜t+1,t⋯op×mC˜t+2,tA˜t+1,tB˜t,tC˜t+2,tB˜t+1,tD˜t+2,t⋱⋮⋮⋱⋮C˜t+Hp,t∏t+Hp−1i=t+1t+HpA˜i,tB˜t,tC˜t+Hp,t∏i=t+2t+Hp−1A˜i,tB˜t+1,t⋯C˜t+Hp,t∏i=t+Hc+A˜i,tB˜t+Ht−1,t,ΔUt=ΔμttΔμt+1t⋮Δμt+Hct,Φt=d˜ttd˜t+1t⋮d˜t+Hp−1t,Λt=et+1t⋮et+Hpt .

The first term is used to predict the difference between the output of the time range *H*_*p*_ and the reference output. The second term is used to control the increment of *H*_*c*_ within the control time range. The third term is used to control the size of the system's control variable in the control time range *H*_*c*_. However, because the system is constantly changing, the optimization objective function that satisfies the constraints is not always able to obtain the best solution in the control cycle [15]. Therefore, it is necessary to add a relaxation factor to the optimization objective function so that when there is no optimal solution during the control period, the optimal solution is replaced with the suboptimal solution obtained from the system, and a feasible solution appears.

### 3.4. Overall Framework of Sports Intelligent Learning Sensor Network

The entire limb rehabilitation monitoring system includes ZigBee-based network equipment and PC or mobile phone. The system is simple in composition and can be easily used by nontechnical personnel. The above-mentioned ZigBee network equipment includes the coordinator system node and the terminal nodes of various motion sensors and pressure sensors configured on the human body, as shown in Figure 1 as the framework of the limb rehabilitation monitoring system.

The entire limb rehabilitation monitoring system includes four parts: ZigBee terminal node, ZigBee coordinator, PC side, and server side. The ZigBee terminal node part includes basic functional modules such as power supply part, pressure and motion sensor part, radio frequency circuit, etc. ZigBee coordination: The device contains interfaces such as radio frequency circuits, serial ports, LEDs, buttons, and other peripheral circuits [16]. The part on the PC side contains the PC and is a combination of the gateway part. It can convert the network protocol on the PC side and send data to the PC. The server side mainly uses the database on the server to remotely save the data processed on the PC.

## 4. Feedback Delay of Intelligent Sports Learning System

### 4.1. Design of Intelligent Sports Learning System

In this article, we combine several smart education theories with school sports rules, combine the results of applying psychological theories in the field of education, integrate several smart education concepts into the physical education process, and then conduct group experiments. The characteristics of student intelligence have formed a model of “diversified sports” with different educational forms, contents, methods, different assessments and evaluations, and student-oriented teaching methods (Table 1). The new diversified intelligent sports teaching model adopted in physical education has achieved better teaching results than before.

The teaching process emphasizes teachers' leadership and students' subjectivity. In the training, through the teacher's teaching, students understand the theoretical basis and technical essence of the technology. Through examples, students can learn the technical foundation and motivate them to learn through organized learning [17]. In addition to theoretical knowledge, students should also develop practical skills, combine classroom learning with humanistic teaching practice, create more internship opportunities, and improve students' ability to deal with and solve problems. Use group project cooperation to promote students' collective spirit. Teachers and students often send “information” and provide feedback in order to improve teachers' control of the teaching process and improve the learning effect. For students with individual differences, teachers need to provide more guidance and communicate with groups. In this way, everyone can make progress together and enhance the cohesion of the class. According to the objectives of the course overview, this paper uses the theory of multiple intelligences to divide the course into three levels (basic, extension, and Research). The three levels are divided into three levels: standard level (A), development level (B), and professional level (C).

According to students' different abilities and their different interests and aspirations, we can choose the education content especially. The content of education should not be invariable but should be updated with the pace of innovation and modern times. Teachers can practice some interesting games in class, which stimulate students' interest and learning enthusiasm. At the same time, we consciously create an environment and conditions for students to describe themselves so as to develop their expressiveness and skills on the spot according to various teaching contents.

The traditional teaching method is very simple and can not meet the different needs of all students, and the teaching method is limited. However, multiple teaching methods can help solve this problem. In the theory of multiple intelligences, the development of intelligence has its own way, and everyone has different combinations of intelligence. These characteristics lead to differences among students. Under the guidance of the theory of multiple intelligences, physical education should pay more attention to human orientation, respect students' learning style, and intelligence characteristics, and design appropriate teaching methods according to each characteristic [18]. Through the teacher's technical explanation and action demonstration, as well as the students' group practice, each student can carry on the practical application, not only knowing how to learn but also knowing how to teach. Students learn in the atmosphere of mutual communication, encouragement, cooperation, exhibition, and competition, which can not only let students express themselves but also deepen their memory of other students' technologies [19]. The observer's job is to compare the practitioner's behavior with the teacher's demonstration behavior, explain the nature of the behavior, and provide useful feedback to the practitioners. This teaching method not only increases students' interest in learning but also speeds up the formation of technical behavior and shortens the learning cycle of technical action. This not only helps to prove students' subjectivity but also paves the way for the development of students' innovation and practical skills.

### 4.2. Design of Intelligent Physical Education Learning Experiment

Before the experiment, the students in two classes were tested for physical quality and basic skills, and the two teaching methods were compared according to the teaching results of the two teaching methods.  Table 2 shows the teaching methods of physical education with multiple intelligence.

The first stage: through appropriate teaching methods to promote students' intelligence. Using multimedia technology or topic analysis to stimulate students to obtain three-dimensional multilevel experience. The second stage: to participate in hands-on activities to develop and expand students' intelligence and improve their practical skills. The third stage: under the guidance of different intelligence theories, the correct choice of education strategies so that students can actively participate in and fully demonstrate their subjectivity [20]. The fourth stage: the transition stage of the learned skills. The fifth stage: provide various assessment toolboxes, carry out intelligent assessments, and test physical fitness and basic skills of experimental class and control class. The experiment first performs the pretest and then uses the pretest standard as the test standard. According to the evaluation content of the national sports standard students' physique standard, the preliminary test index is determined, and on the basis of this evaluation, a systematic comparative study is carried out (see Table 3).

### 4.3. Research on Time-Delay Control

Generally speaking, chaos control includes two aspects: when the chaos phenomenon causes the system to collapse or is not the expected state, the control system returns to the periodic state. When we expect the system to produce chaos to achieve our ideal output, the control system will produce chaos, even a specific chaotic orbit.

Chaos has a very strong dependence on the initial value. The disturbance in the process of motion or the change of system parameters will also lead to chaos. The phenomenon, which is very different from the periodic state caused by the change of state value, can also be used to control the chaos. All kinds of chaos control methods discovered and studied by predecessors are the angle of adjusting a certain control parameter. So far, there are a variety of control strategies and modes. According to the characteristics of each system and the different control effects required by different characteristics, the following control methods are summarized. Up to now, all control strategies can be classified into these categories: the first category belongs to the category of parameter perturbation, and the typical one is the OGY method. It is also the first method proposed to control the chaos. The second one belongs to the feedback type, which takes the time delay feedback method as a typical example, and takes the output part of the system as the feedback control variable to directly act on the input of the control system. The third type is the nonfeedback type, which directly controls the state variables, such as the parametric resonance perturbation method, external noise control method, and so on. The fourth is adaptive control, which tends to be an intelligent control algorithm. In the end, the PID parameter method based on inverse Nyquist delay is proposed.

### 4.4. Simulation Results

The delay is simulated by the transport delay module. After the ramp signal is compared with the feedback signal, the sign function is used to filter the output NMOS driving voltage. Above, the gain stability range of *T*/4 delay is obtained by the PID parameter tuning method with time delay. Next, the motion of the system with different time delays and different gains is visually observed by the simulation diagram, and the gain stability range obtained by the parameter tuning method with time delay is verified.

Corresponding to the simulation analysis, firstly, change the input, take *t*/4 as the delay factor, take 8.4 as *K*_2_, and change from 15 V to 32 V excessively. The simulation diagram is shown in Figure 2. Take 15 V, 23 V, 24 V, 26 V, 28 V, and 32 V as the simulation diagram.  Figure 3(a) shows the change of control signal, and Figure 3(b) shows the phase change diagram.

When Vin increases to more than 40 V, there is no complete chaos phenomenon. When Vin is between 25.28 V and 38 V, double period and steady-state crossover appear, as shown in Figure 2.

First, select the delay factor *γ*, take *T*/16, *T*/8, *T*/4, *T*/2, *T*, 2*T* for horizontal comparison, and then take *k*_2_ as a different value for vertical comparison as shown in Figure 4.

When *γ* = *T*/8, take Vin as 33 V and get the variation of V0 with 2*k*, as shown in Figure 5.

The value comparison is shown in Table 4.

It can be seen that when the delay is *T*/16, the control effect is not ideal. When the delay is increased to *T*/4, the control effect is better. When *K*_2_ is set between [5, 30], the motion is mostly in a single periodic state. When the delay is *T*/8, the control effect of *K*_2_ is better when the value of [7, 8] is only used. The effect of each delay time and the value of K_2_ is shown in Table 5.

In the time delay feedback control experiment of the chaotic phenomenon of the circuit caused by the input change and the capacitance change, we can find that when the delay time is *T*/16, *K*_2_ selects certain points, and the system adjustment effect is general; when the delay time is *T*/8, *K*_2_ has a better system adjustment effect at certain points; when the delay time is *T*/4, *K*2 has a wider value range, and the system adjustment effect is better in a certain range for the chaos caused by input, capacitance, and frequency changes; When the delay time is *T*/2, the adjustment of the results at different inputs is inconsistent, and the result adjustment tends to be inconsistent, with a large error; after the delay time is increased to *T*, the system output results are obviously dispersed, and the error is aggravated; At 2*T*, chaos and bifurcation are more severe. From this experiment, we can see that the delay feedback factor is *T*/4, and the chaos control effect is better.

## 5. Conclusion

The application of multiple intelligences theory in college physical education can improve the shortcomings under the guidance of traditional intelligence theory, improve the content provided in traditional courses, and organize the courses and training of body movement intelligence. The educational model based on the theory of multiple intelligences expands the scope of curriculum” “Multiple Intelligences Education” and “multiple intelligences teaching” focus on the curriculum training of seven bits of intelligence. At the same time as intelligent training, we can not ignore the cultivation of intelligence. We pay attention to students' personality and learning styles and adopt more suitable teaching methods according to various intelligent characteristics. This is not only in line with the essence of quality education but also lays a firm foundation for a new round of curriculum reform and promotes the practice of quality education to be more practical. Research on predictive control algorithm of the linear time-varying model. In view of the complexity of the nonlinear model and nonlinear constraints will increase the difficulty of solving predictive control problems in a nonlinear model, this paper introduces how to transform a nonlinear time-varying system into a linear time-varying system and how to derive predictive control algorithm formula for a linear time-varying predictive model, and how to transform the optimization problem of LTV-MPC into a practical standard quadratic programming problem that can be solved by computer.

## Figures and Tables

**Figure 1:** Schematic diagram of limb rehabilitation monitoring system framework.

**Figure 2:** The output of the circuit when the input is increased after the two-cycle state.

**Figure 3:** The control signal and phase diagram change at 8.4.

**Figure 4:** When delaying *T*/16, the effect of different values of *K*_2_ under 33 V input.

**Figure 5:** When delaying *T*/8, the effect of different values of *K*_2_ under 33 V input.

**Table 1:** Design framework of multiple teaching mode.

Multiple physical education teaching mode			
Form	Content	Method	Evaluation
1. Combination of theory and practice	1. Targeted	1. Teacher leadership method	1. Normal performance assessment
2. Combination of teachers and students	2. Innovative	2. Model demonstration and encouragement method	2. Technical performance assessment
3. Combination of exercise and practice	3. Specific attraction	3. Group cooperative learning method	3. Theoretical performance assessment
4. Combination of group practice and group practice	4. Outstanding self-sufficiency	4. Teaching competition method	4. Teaching performance practice assessment
	5. Content rich and selective	5. Role switching method	

**Table 2:** The teaching steps of multiple intelligences in Physical Education.

Learning phase	The first stage	The second stage	The third phase	The fourth stage	The fifth stage
Teaching task	Awaken intelligence; through various effective teaching methods, activate students' various intelligence abilities	Enter special practice activities to improve students' various bits of intelligence and promote the improvement of professional learning ability	Give full play to students' subjective initiative and use relevant teaching strategies to create opportunities for students to think about and learn actively	In the skill transfer stage, the positive transfer of strong intelligence is promoted through flexible and diverse teaching methods, and the weak intelligence group is improved.	Provide diversified multidimensional evaluations and conduct various assessment tests for experimental classes and control classes

Specific implementation method	Broadcast sports programs and popularize sports culture knowledge through multimedia so that students can effectively stimulate their hobbies and interests in sports. (Use 4 class hours)	Use group exercises, team competitions, special games, various special combination exercises, etc., to integrate the ability of body movement intelligence into sports learning to improve learning initiative (20 class hours)	Cultivate interpersonal intelligence, cultivate team spirit; develop students' intelligence through sports practice activities, actively guide students, and improve their learning (10 class hours)	Show the personality of the student. In the education process, the teacher actively guides and encourages the student (15 class hours)	Emphasizes the intelligence of self-understanding, and summarizes the content reflected in education and learning, and provides students with various assessment experiences (5 class hours)

**Table 3:** Results of body shape and quality test of two groups before experiment.

Test content	Experimental group *n* = 30	Control group *n* = 30	*t*	*P*
Age/year	20.98 + 0.88	21.06 ± 0.65	0.78	>0.05
Height/m	1.70 ± 0.10	1.72 ± 0.32	1.00	>0.05
Weight/kg	62.50 ± 4.60	64.8 ± 5.86	0.96	>0.05
Vital capacity (ml)	3218 ± 546	3198 ± 538	0.12	>0.05
Step test	49 ± 5	52 ± 5	0.22	>0.05
50 m run (s)	9.16 ± 1.0	8.90 ± 1.12	0.34	>0.05
Standing long jump (m)	1.91 + 0.86	1.95 + 1.15	0.45	>0.05
Grip strength and body mass index (male)	62 ± 5	59 ± 5	0.34	>0.05
Sit-ups (female)	25 ± 5	24 ± 4	0.05	>0.05

**Table 4:** When input causes chaos, the comparison table when *γ* and 2*k* have different values.

*K*_2_/*t*	*T*/16	*T*/8	*T*/4	*T*/2	*T*	2*T*
[1, 70]	Select the appropriate K_2_ control effect is general	Choose the appropriate K_2_ control effect is better	Choose the appropriate K_2_ control effect is better	Select the appropriate K_2_ control effect is general	The control effect is poor	The control effect is poor

**Table 5:** When the capacitance causes chaos, the comparison table when *γ* and *K*_2_ have different values.

*k*_2_/*T*	*T*/16	*T*/8	*T*/4	*T*/2	*T*	2*T*
[1,70]	Select the appropriate K_2_ control effect is general	Choose the appropriate K_2_ control effect is better	Choose the appropriate K_2_ control effect is better	Select the appropriate K_2_ control effect is general	The control effect is poor	The control effect is poor

## Data Availability

The data used to support the findings of this study are available from the corresponding author upon request.

## References

[1] Qin H. K.W. (2018). Research on 020 platform and promotion algorithm of sports venues based on deep learning technique. *International Journal of Information Technology and Web Engineering*.

[2] Khan A. S., Khan F. U. (2021). A survey of wearable energy harvesting systems. *International Journal of Energy Research*.

[3] Martin T., Jovanov E., Raskovic D. Issues in wearable computing for medical monitoring applications: a case study of a wearable ECG monitoring device.

[4] Redmon J., Farhadi A. YOLO9000: better, faster, stronger.

[5] Matina R. M., Rogol A. D. (2011). Sport training and the growth and pubertal maturation of young athletes. *Pediatric Endocrinology Reviews*.

[6] Chanjira P., Permpoonsinsup W., Tunyasrirut S. (2018). Metaheuristic optimization algorithm for PI control buck-boost converter based on wind turbine. *International Journal of Pure and Applied Mathematics*.

[7] Pakdeeto J., Chanpittayagit R., Areerak K., Areerak K. (2017). The optimal controller design of buck-boost converter by using adaptive Tabu search algorithm based on state-space averaging model. *Journal of Electrical Engineering and Technology*.

[8] Lasota A., Mackey M. C. (1994). Chaos, fractals, and noise. *Stochastic aspects of dynamics*.

[9] Vandenbergh F., Engelbrecht A. (2006). A study of particle swarm optimization particle trajectories. *Information Sciences*.

[10] Pistorius J., Hutton M. Placement rent exponent calculation methods, temporal behaviour and FPGA architecture evaluation.

[11] Mikki S. M., Kishk A. A. (2007). Physical theory for particle swarm optimization. *Progress in Electromagnetics Research*.

[12] Trelea I. C. (2003). The particle swarm optimization algorithm: convergence analysis and parameter selection. *Information Processing Letters*.

[13] Kaptanoglu S. Power and the future FPGA architectures.

[14] DeHon A. Balancing interconnect and computation in a reconfigurable computing array (or, why you don’t really want 100% LUT utilization).

[15] Wang L., Xiong Y., Wang Z. Temporal segment networks: towards good practices for deep action recognition.

[16] Śmieja M. (2018). ZigBee phase shift measurement approach to mobile inspection robot indoor positioning techniques. *Diagnostyka*.

[17] Hagenbuchner M., Cliff D. P., Trost S. G., Van Tuc N., Peoples G. E. (2015). Prediction of activity type in preschool children using machine learning techniques. *Journal of Science and Medicine in Sport*.

[18] Fischer E., Hänze M. (2019). Back from “guide on the side” to “sage on the stage”? Effects of teacher-guided and student-activating teaching methods on student learning in higher education. *International Journal of Educational Research*.

[19] Nasser-Abu Alhija F. (2017). Teaching in higher education: good teaching through students’ lens. *Studies In Educational Evaluation*.

[20] Casado M. (2000). Teaching methods in higher education: a student perspective. *Journal of Hospitality and Tourism Education*.

